The article "Distinct gene expression profiles associated with clinical outcomes in patients with ovarian clear cell carcinoma and high-grade serous ovarian carcinoma" was published in 2020. Journal: J Ovarian Res.

# Distinct gene expression profiles associated with clinical outcomes in patients with ovarian clear cell carcinoma and high-grade serous ovarian carcinoma

**DOI:** 10.1186/s13048-020-00641-8

**Published:** 2020-04-15

**Authors:** Huimei Zhou, Qian Liu, Xiaohua Shi, Yue Liu, Dongyan Cao, Jiaxin Yang

**Affiliations:** 1 Department of Gynaecologic Oncology, Peking Union Medical College Hospital, 1 Shuaifuyuan, Dongcheng-qu, Beijing, People’s Republic of China; 2 Department of Pathology, Peking Union Medical College Hospital, Beijing, People’s Republic of China

**Keywords:** Ovarian clear cell carcinoma, Gene expression profiles, High-grade serous ovarian carcinoma, Outcome

## Abstract

**Background:**

Ovarian clear cell carcinoma (OCCC) is the second most common ovarian cancer after serous carcinoma in Southeast Asia. OCCC has a more unfavourable clinical outcome due to a poor response to platinum-based chemotherapy compared with serous carcinoma. The identification of biomarkers related to the prognosis of OCCC is critically important for an improved understanding of the biology that drives OCCC progression and leads to poor outcomes. To detect differences in gene expression profiles between OCCC and high-grade serous ovarian carcinoma (HGSOC), twelve patients with OCCC and twelve patients with HGSOC were recruited in whom the pathological diagnosis was confirmed on surgically resected specimens.

**Results:**

Compared with HGSOC, OCCC has 609 differentially expression genes, and 199 are significantly different (*P* < 0.05). These genes are involved in the cell cycle, apoptosis, DNA damage repair, the PI3K pathway and so on. There were 164 differentially expressed genes in the PI3K pathway. There were 35 overexpressed genes in OCCC, while there were 12 overexpressed genes in HGSOC. Among these differentially expressed genes, we found that the MET gene and the CCNE1 gene were overexpressed in OCCC and associated with a worse prognosis.

**Conclusions:**

In conclusion, there are many differentially expressed genes in OCCC and HGSOC, which indicates that the two kinds of tumours differ greatly in tumourigenesis and provides a theoretical basis for targeted therapy in the future. Further studies need to be performed to clarify the association of the differentially expressed genes with the unfavourable prognosis in OCCC.

## Background

Different histological subtypes of epithelial ovarian cancer have different molecular characteristics and clinical prognosis [1]. Ovarian clear cell cancer (OCCC) accounts for 10% of epithelial ovarian cancers and is known to be typically resistant to platinum-based chemotherapy and associated with a poorer prognosis than the more common serous subtype [2]. Although the carcinogenic mechanism and chemoresistance of OCCC are still unclear, several genetic changes have been extensively studied. Compared with HGSOC, OCCC is usually negative for p53 mutations, and the frequency of breast cancer 1 or 2 (BRCA1/2) mutations is low (6.3%) [3, 4]. Higher frequencies of AT-rich active domain 1A (ARID1A) and phosphatidylinositol-4,5-diphosphate 3-kinase catalytic subunit alpha (PIK3CA) mutations (36%) have also been observed in OCCC patients [5, 6]. Therefore, further search for new tumour markers of chemoresistance and the development of new therapeutic targets are needed to help identify the mechanism of OCCC and for the effective clinical management of OCCC. Our study aimed to identify the molecular landscape of OCCC compared with HGSOC using the NanoString® PanCancer 770 gene Pathway Panel to evaluate changes in RNA expression and their association with clinical outcomes.

## Patients and methods

### Patient data and clinicopathological features (Table 1)

Medical records of women with a diagnosis of OCCC and HGSOC patients who were treated between December 2013 and April 2017 at Peking Union Medical College Hospital were reviewed retrospectively. This study was approved by the ethics committee of PUMCH. Clinical and pathologic data were obtained from the medical records. A total of 24 patients with OCCC and HGSOC without preoperative chemotherapy whose tumours were surgically resected and pathologically confirmed were recruited for this study.

**Table 1:** Clinical characteristics of twenty-four patients

Clinical characteristic	OCCC (*N* = 12)	HGSOC (*N* = 12)
Age (years)	47 (32 ~ 62)	57.6 (39 ~ 75)
Stage		
Ic	1	1
IIb	1	0
IIIa	1	0
IIIb	1	0
IIIc	7	9
IVb	1	2
Disease status at the last follow-up		
Alive with disease	6	7
Dead with disease	6	5

Details of surgery were collected from the operative records. Optimal cytoreduction was defined as < 1 cm of residual disease at the time of cytoreductive surgery. All of the patients were followed up every 3 months for the first 3 years, every 6 months for the following 2 years, and then once the following year. Oncologic outcomes were evaluated by a gynaecologic oncologist. Clinicopathological characteristics of these patients, such as age, the International Federation of Obstetrics and Gynecology (FIGO) stage, treatment regimens, recurrence, progression-free survival (PFS), and overall survival (OS), were reviewed.

### NanoString nCounter analysis

Formalin-fixed, paraffin-embedded tumour samples were identified, and specimens were reviewed for a pathologic diagnosis and dissected if necessary to ensure that ≥90% of the sample represented the tumour. Samples were processed for analysis on the NanoString nCounter Flex system using the 770 gene PanCancer Pathways Plus panel (606 critical genes from 13 canonical cancer pathways, 124 cancer driver genes, and 40 reference genes) per the manufacturer’s instructions (NanoString Technologies, Seattle, WA).

NanoString expression analysis identifies the differentially expressed genes in the selected patient specimens. The histological specimens of the selected cases required an effective area > 1.5 * 1.5 cm and 3 ~ 5 10 μm wax rolls, and puncture specimens increased the number of wax rolls according to the tissue area. The experimental procedure included total RNA extraction, sample QC, overnight hybridization, hybrid product elution purification, sample plate preparation, sample plate scanning, and output.

### Statistical analysis

NanoString data and pathway analyses are described above. Genetic polymorphisms and clinicopathological parameters in OCCC and HGSOC were assessed using Pearson’s chi-square test or Fisher’s exact test. The univariable survival analysis was performed by the generation of Kaplan-Meier curves, and differences between the groups were assessed using the log-rank statistic. SPSS v24.0 (SPSS, Inc., Chicago, IL, USA) was applied for all analyses. *p* values < 0.05 were considered significant.

## Results

### Clinical characteristics

Between December 2013 and April 2017, twelve patients with OCCC and twelve patients with HGSOC received treatment at PUMCH. All patients were treated with primary debulking surgery/comprehensive staging and platinum-based adjuvant chemotherapy postoperatively. The baseline clinical data of all patients are shown in Table 1. The average follow-up time of 24 patients was 27.1 months (4.2 ~ 49.6 months), and the average recurrence interval was 6.2 months (1 ~ 19.7 months).

### NanoString expression analysis identifies differentially expressed genes between OCCC and HGSOC

We performed NanoString expression analysis with the NanoString nCounter Flex system using the 770 gene PanCancer Pathways Plus panel (606 critical genes from 13 canonical cancer pathways, 124 cancer driver genes, and 40 reference genes) to compare OCCC and HGSOC tumour tissue in the patient cohort described in Table 1.

Compared with HGSOC, OCCC has 609 differentially expressed genes, and 199 were significantly different (*P* < 0.05). The pathways involved included the cell cycle, apoptosis, chromatin modification, DNA damage repair, driver genes, the Hedgehog, JAK-STAT, MAPK, Notch, PI3K, Ras, TGF-beta, and Wnt pathways and transcriptional misregulation (Fig. 1).

**Fig. 1:** Expression of different genes between the OCCC and HGSOC groups (Volcano map)

### The PI3K pathway shows more dominant alterations in OCCC compared with HGSOC

Cancer-related pathways may serve as potential targets for therapeutic intervention. In this analysis, we identified 164 differentially expressed genes in the PI3K pathway. A notable observation was the significantly higher expression of 35 genes in the tumour tissue of OCCC compared with HGSOC and the significantly lower expression of 12 genes in the tumour tissue of OCCC compared with HGSOC (Fig. 2). Among these differentially expressed genes, PI3K pathway analysis revealed that the MET gene and the CCNE1 gene were associated with worse clinical outcomes. These two genes appeared to be more highly expressed in OCCC compared to HGSOC (Fig. 3 and Fig. 4).

**Fig. 2:** Related differentially expressed genes involved in the PI3K pathway (heatmap)

**Fig. 3:** Patients with a high MET level have a poor prognosis (*P* = 0.012)

**Fig. 4:** Patients with a high CCNE1 level have a poor prognosis (*P* = 0.030)

## Discussion

Treatment regimens for OCCC and HGSOC are the same at present; however, the clinical outcome between them is very different. Many studies have reported that these two kinds of ovarian cancer have different origins [6, 7]; therefore, new attractive therapeutic targets will focus on differences in the genetic expression between the two cancers. Due to the poor prognosis and chemotherapy resistance of OCCC patients, a reliable genetic diagnosis and targeted therapy are beneficial to patients with rare types of ovarian cancer. Clinical observation and genomic testing are both necessary in the exploration. Mutations in PIK3CA (32–33%), ARID1A (46%), KRAS and BRAF are very common in the somatic mutation of OCCC [8, 9]. The differentially expressed genes between these two subtypes of ovarian cancer are involved in multiple cancer pathways, including the cell cycle, apoptosis, chromatin modification, DNA damage repair, driver genes, the Hedgehog, JAK-STAT, MAPK, Notch, PI3K, Ras, TGF-beta, and Wnt pathways, and transcriptional misregulation. Furthermore, the PI3K pathway was one of the top pathways associated with these differentially expressed genes. Currently, targeted therapy for this pathway provides many new alternative options for the therapy of OCCC patients with a poor prognosis and treatment dilemma.

The MET proto-oncogene is located at chromosome 7q31 and encodes MET kinase, which is composed of three functional domains: the ligand-binding domain, the regulatory juxtamembrane domain, and the receptor tyrosine kinase domain [10]. In tumour cells, MET can be activated in a ligand-independent manner by mutating, amplifying or overexpressing the MET gene [11]. The MET signalling pathway is involved in processes of tumourigenesis, such as tumour proliferation, protection from apoptosis, angiogenesis, and motility [12]. Studies have confirmed that c-MET activation is associated with adverse clinical outcomes in lung, breast, stomach, kidney, and head and neck cancers [13, 14].

In EOC, MET is overexpressed in 7–27% of the population and is associated with progression and adverse outcomes of ovarian cancer [15]. Yamamoto et al. found that MET overexpression and gene amplification are ubiquitous in ovarian clear cell adenocarcinoma, with frequencies as high as 22–24% [16]. The MET proto-oncogene in OCCC participates in tumourigenesis through gene amplification. On the other hand, this change is extremely rare in nontransparent cell histological subtypes of ovarian cancer (i.e., serous, endometrioid, and mucinous adenocarcinoma). Recently, studies have reported that the c-MET amplification rate in OCCC is as high as 37.0% and is associated with poor survival [17]. MET overexpression is associated with a poor prognosis in patients with OCCC. Kim HJ et al. investigated the therapeutic effects of c-MET inhibitors on OCCC. The results showed that the inhibition of c-MET by c-MET inhibitors (SU11274 or crizotinib) significantly reduced OCCC cell proliferation and increased apoptosis. In vivo experiments confirmed that c-MET inhibitors can significantly reduce the tumour weight of the RMG1 cell xenograft model in vivo and the OCCC PDX model [10].

Compared with ovarian serous or endometrioid carcinoma, OCCCs have obvious chemotherapy resistance and poor prognoses. Previous studies have shown that stage I/II OCCCs have a better prognosis than HGSOC, while stage III/IV OCCCs have a worse prognosis than HGSOCs [18]. The combination of Met and CD44 and CD47 may promote the progression of OCCCs [19]. OCCCs with Met amplification may have worse clinical outcomes. Therefore, alternative therapies for OCCCs, such as molecular targeted therapy, are urgently needed. It is difficult to target the deletion of ARID1A, which often cooperates with the P53 gene. Therefore, Met is considered a good candidate for targeted therapy because of its high frequency of amplification and its high mutation specificity in OCCCs.

In this study, differentially expressed genes between OCCC and HGSOC and those associated with a poor prognosis were analysed by NanoString. The expression of MET was significantly different between OCCC and HGSOC; it was more highly expressed in OCCC compared to HGSOC. This is consistent with the results of previous studies. There was a significant correlation between high MET expression and good OS and between low MET expression and poor OS. The results should be confirmed further because of the relatively short follow-up time. It is still necessary to further verify the effects of the MET gene on the occurrence, development and drug resistance of OCCC at different levels and provide a more theoretical basis for the treatment of OCCC with the MET gene as a target.

The CCNE1 gene encodes the cell cycle E1 protein, which promotes the activity of cyclin-dependent kinase-2 (Cdk2) and plays an important role in regulating the transition from G1 to S phase of the cell cycle [20]. One study reported that the CCNE1 gene also has direct action in triggering DNA replication and maintaining genomic stability [21]. Several studies have reported that CCNE1 gene amplification or protein upregulation is associated with higher tumour grades and a worse clinical outcome in a variety of cancers [22, 23]. CCNE1 overexpression is observed in ovarian high-grade but not low-grade serous carcinomas. Exome sequencing identified 26% of OCCC patients with amplifications in the *CCNE1* locus whose copy number gain was previously shown to be correlated with increased protein expression and associated with a worse outcome [24]. These results suggest the importance of CCNE1 in the progression of OCCC and support cyclin E1 as a possible therapeutic target in OCCC. In our study, we found that CCNE1 was more strongly overexpressed in OCCC patients than in HGSOC patients, which seems to be correlated with worse outcomes. These results suggest the importance of CCNE1 in the progression of OCCC and support cyclin E1 as a possible therapeutic target in OCCC.

As already stated, OCCC is the second most common ovarian cancer after serous carcinoma and represent 26% of ovarian cancer in Southeast Asia [3]. However, fewer molecular targets have been identified for OCCC compared with HGSOC. To the best of our knowledge, we present here the series with a distinct gene expression identification for these two histotypes of Chinese ovarian cancer for the first time. We found that MET and CCNE1 maybe play tumorigenesis roles in OCCC. These genes could be used as biomarkers and therapeutic targets for OCCC. Additional functional analysis for these genes is necessary to reveal new targets of OCCC.

We would like to acknowledge some of the limitations of the study. This study was retrospective and performed on a small but relevant patient population in that most of patients were in advanced stage at need population. Despite this limitation, these findings present an opportunity to rationally approach future clinical trials in the treatment of OCCC.

## Conclusions

In general, the system identification of differentially expressed genes in OCCC and HGSOC will enlighten us on the differences in tumorigenesis and provides a theoretical basis for targeted therapy of OCCC in the future. Further studies need to be performed to clarify the association of the differentially expressed genes with the unfavourable prognosis in OCCC. The present and future results will be applied to the development of potential diagnostic and therapeutic options for OCCC.

## Data Availability

All data generated or analysed during this study are included in the published article.

## Abbreviations

CI: Confidence interval
FIGO: International Federation of Obstetrics and Gynecology
HR: Hazard ratio
IRB: Institutional Review Board
OCCC: Ovarian clear cell carcinoma
OS: Overall survival
PFS: Progression-free survival
